# Molecular Cloning and Docking of *speB* Gene Encoding Cysteine Protease With Antibiotic Interaction in *Streptococcus pyogenes* NBMKU12 From the Clinical Isolates

**DOI:** 10.3389/fmicb.2018.01658

**Published:** 2018-08-07

**Authors:** Natesan Balasubramanian, Govintharaj Varatharaju, Vellasamy Shanmugaiah, Karuppiah Balakrishnan, Mandayam A. Thirunarayan

**Affiliations:** ^1^Department of Immunology, School of Biological Sciences, Madurai Kamaraj University, Madurai, India; ^2^Department of Microbial Technology, School of Biological Sciences, Madurai Kamaraj University, Madurai, India; ^3^Department of Microbiology, Apollo Hospitals, Chennai, India

**Keywords:** antibiotic resistance, gene cloning, cysteine protease, *Streptococcus pyogenes*, virulence factors, docking analysis

## Abstract

*Streptococcus pyogenes* causes a variety of diseases ranging from mild diseases to severe invasive infections which result in significant morbidity and mortality. This study focuses on the antibiotic resistance of *S. pyogenes* and their interaction with cysteine protease. Around 36 beta-hemolytic isolates were collected from the clinical lab, of which seven isolates (19.4%) were identified as *Streptococcus pyogenes*. One of the seven isolates was collected from a urinary tract infection, which was identified by antibody agglutination and MALTI-TOF-MS, and it is designated as *S. pyogenes* NBMKU12. Around 8.3 to 66.6 % of the isolates were found to be resistant to one or more antimicrobial agents, especially, penicillin-G resistance was exhibited by 29.1% of the isolates. In the NBMKU12 isolate, the beta lactem (*TEM*) gene was detected among the 13 antibiotic genes for which it was tested. Furthermore, when analysis for presence of 13 virulence genes were carried out in NBMKU12 isolate, only *speJ* and *speB* were detected. The *speB* (streptococcal pyrogenic exotoxin B) encoding cysteine protease gene was cloned. This was followed by performing DNA sequencing to understand the putative cysteine protease interaction with antibiotics, inhibitors, and substrate. The *speB* gene consists of 1197 nucleotides and encodes a protein with multiple domains, including a signal peptide (aa 1–22), an inhibitor region (aa 27–156), and a catalytic cysteine domain (aa 160–367). The signal peptide cleavage site is predicted between Ala22 and Asn23. The putative 398 amino acid residues were found to have a theoretical pI of 8.76 and a molecular mass of 43,204.36 Da. The tested culture supernatants of NBMKU12 isolate exhibited the proteolytic activity against casein, papaya and pineapple used as substrates. The proteolytic activity suggests the expression of speB gene. Molecular docking analysis of cysteine protease showed that erythromycin (bond length 2.41 Å), followed by chloramphenicol (2.51 Å), exhibited a strong interaction; while penicillin-G (3.24 Å) exhibited a weak interaction, and this factor could be considered as a cause for penicillin-G resistance. The present study contributes to a better understanding of *speB* gene encoding cysteine protease, antibiotic resistance, and their interaction in the isolate, *S. pyogenes* NBMKU12. The antibiotics and cysteine protease interaction study confirms the resistance or sensitivity of *S. pyogenes*. Hence, it could be hypothesized that the isolate NBMKU12 is resistant to most of the tested antibiotics, and this resistance might be a cause for mutation.

## Introduction

*Streptococcus pyogenes* (Group A Streptococci) is the most widespread pathogenic bacteria that infects children and adolescents (Brook and Dohar, 2006). It causes a wide range of infections from pharyngitis to severe systemic diseases, such as necrotizing fasciitis or streptococcal toxic shock syndrome (STSS), and post-infection complications (Cunningham, 2000; Pires et al., 2012). Moreover, *S. pyogenes* causes extensive cutaneous infections ranging from superficial cellulitis to severe cellulitis, and even life-threatening pyoderma (Sumitomo et al., 2018). Group A streptococci (GAS) phage-associated pyrogenic exotoxins or superantigens (Jing et al., 2006) have been shown to cause severe diseases such as scarlet fever, rheumatic fever, and rheumatic heart diseases (Rato et al., 2010).

Most of the *S. pyogenes* strains are susceptible to penicillin (Bassetti et al., 2000), and hence penicillin is universally recommended for treatment of *S. pyogenes* infections (Bowen et al., 2012). However, macrolides are used as an alternative in penicillin-allergic patients (Camara et al., 2013). Further, increased macrolide-resistance and asymptomatic oropharyngeal colonization of *S. pyogenes* have been reported in different countries (Felmingham et al., 2004; Chang et al., 2010). In recent years, an increase of up to 50% in streptococci resistance to penicillin has been observed (Nunes et al., 2005). Recent surveillance studies have shown temporal changes in drug-resistant streptococci, predominantly due to environmental factors, and this could be a major reason for drug-resistant strains causing pediatric and adult diseases (Nunes et al., 2005; Camara et al., 2013).

*Streptococcus pyogenes* are primarily identified using the antibiotic bacitracin to which it is susceptible. This acts as the factor for differentiating beta-hemolytic streptococci in human infections (Facklam, 2002). However, recently isolated clinical isolates are found to be resistant to bacitracin (Perez-Trallero et al., 2007). Keeping the important development of streptococcal resistance in mind, we have studied the collection of human isolates of *S. pyogenes* for their genetic determinants of resistance to ampicillin, penicillin-G, tetracycline, chloramphenicol, and vancomycin. The present research work has been carried out to understand the antibiotic resistance mechanism in the NBMKU12 isolate and its putative cysteine protease interaction with selected antibiotics, substrates, and inhibitors. These interaction studies provide vital data concerning virulence genotypes and antibiotic resistance genes of the novel isolate of NBMKU12.

Cysteine proteases consist of 108 different families (Rawlings et al., 2012), and the catalytic residues are present either in the Cys-His or His-Cys order (Richter et al., 2012). In cysteine proteases, the Cys residue acts as the nucleophile agent and the His residue acts as the proton shuttling residue (Cstorer and Menard, 1994). Cysteine proteases are responsible for several biological processes, including degradation of peptides and proteins (Grzonka et al., 2001). Active *speB* encoding cysteine protease cleaves the host extracellular matrix (Kapur et al., 1993), immunoglobulins (Eriksson and Norgren, 2003), and complementary components (Terao et al., 2008). In addition, the cysteine protease has the ability to cleave host proteins (Walker et al., 2007), and this proteolytic activity contributes to the bacterial evasion from the host defense system and systemic dissemination (Nelson et al., 2011). Immunoglobulin G-degrading enzyme and *speB* encoding cysteine protease are the two major cysteine proteases which are secreted by Group A streptococcus (GAS) and involved in host immune suppression (Sumitomo et al., 2013).

The present study also tested the cysteine protease activity in the isolate NBMKU12, using different substrates, to confirm its degradation ability. Here we present the process of *speB* gene detection, its molecular characterization, and putative cysteine protease interaction with antibiotics, inhibitors, and substrate to understand the S. *pyogenes* pathogenesis through a UTI isolate NBMKU12.

## Materials and Methods

### Bacteria Collection and Identification

A total of 36 beta-hemolytic isolates (I-batch) were collected from the Microbiology Laboratory, Apollo Hospitals, Chennai, India. These 36 isolates were isolated from patients receiving medical care in the Apollo Hospitals. The isolates were collected from samples of urine (20), secretions (7), blood (3), and other sources (6). Among the 36 isolates, 7 isolates of *Streptococcus pyogenes*, and 1 isolate of NBMKU12 collected from a patient with urinary tract infection (UTI), were used in this study. The collected isolates were purified and stored at -80°C in sterilized Todd-Hewitt broth with 20% glycerol. The isolates, including NBMKU12, were identified by colony morphology on sheep-blood agar using beta-hemolysis, group A-specific antiserum HiStrep Latex Agglutination Test (HiMedia, India), and MALDI-TOF-MS.

### MALDI-TOF-MS Analysis

The identification of streptococcus by MALDI-TOF-MS system (VITEK MS, BioMérieux, France) was carried out as described earlier (Lartigue et al., 2009). In brief, overnight NBMKU12 fresh colonies were picked from a solid culture, mixed with a CHCA matrix on a conductive target slide, and inserted into the VITEK MS system for performing a rapid automated identification. An *E. coli* calibrator was used for the validation of the similarity analysis. Only those identifications with a score of 99.9% were considered, although a score of >70% was considered acceptable. Identification is based on the signature mass spectrum of each organism that is generated. It was then compared with a validated database of spectra for a range of pathogens. All the spectra were analyzed using a MALDI V3 software package that compares the experimental data with the reference spectra and provides identification.

### Culture Media, Bacterial Growth, and Storage Condition

The solid growth medium was used for culture and colony isolation in Todd-Hewitt Agar, or Colombia agar supplemented with 5% (v/v) sheep blood (HiMedia, India). Liquid cultures were grown in Todd-Hewitt broth supplemented with 1% (w/v) yeast extract, Tryptic Soy broth (HiMedia, India), and incubated at 37° C for 16–18 h. The late exponential phase culture was mixed with 20% sterilized glycerol and maintained at -80°C for further use.

### MIC Test

MIC test was done in E strip on Mueller-Hinton agar with 5% (v/v) sheep blood (HiMedia, India). The plates were incubated for 20–24 h at 37° C. An antibiotic susceptibility test was performed according to the Clinical Laboratory’s Standards Institute (CLSI) guidelines for ampicillin, vancomycin, ceftriaxone, amoxiclav, and chloramphenicol (HiMedia, India).

### Antibiotic Susceptibility Test

Antibiotic susceptibility tests were performed for all isolates of *S. pyogenes* by disk diffusion method. A fresh colony was inoculated in 2 mL of Todd-Hewitt broth with 1% yeast extract and incubated at 37°C for 18–20 h. A 100 μL liquid culture of each isolate was swabbed using sterilized cotton buds on Muller-Hinton agar with 5% sheep blood (HiMedia, India). After the *S. pyogenes* was swabbed, antibiotic disks were placed on the medium. Antibiotic susceptibility was tested against ampicillin (10 mcg/mL), penicillin-G (10 mcg/mL), tetracycline (30 mcg/mL), erythromycin (15 mcg/mL), azithromycin (30 mcg/mL), vancomycin (30 mcg/mL), ceftriaxone (30 mcg/mL), amoxiclav (30 mcg/mL), and chloramphenicol (10 mcg/mL). The plates were incubated at 37°C for 20–24 h. The zone of inhibition was measured, and the results were interpreted according to the Clinical Laboratory’s Standards Institute guidelines (CLSI, 2006).

### Genomic DNA Extraction

The Genomic DNA was isolated using HiPurA bacterial genomic DNA purification kit (HiMedia, India) with slight modifications. Briefly, bacterial cells were grown in 5 mL Todd-Hewitt broth supplemented with 1% yeast extract (w/v) (HiMedia, India), and incubated at 37°C for 16–18 h. The culture was centrifuged at 12000 rpm for 2 min, and the pellet was resuspended in 200 μL lysozyme solution (45 mg/mL). It was then incubated for 30 min at 37°C, followed by the addition of 20 μL Proteinase K (20 mg/mL) and 20 μL RNase mixture, and again incubated at room temperature. Finally, the DNA was eluted with 150 μL of Elution buffer and stored at -20°C or immediately used for polymerase chain reaction (PCR).

### Detection of Virulence Genes in *S. pyogenes*

To check the presence of erythrogenic exotoxins or superantigens in NBMKU12 isolate, the PCR reaction was carried out in single and multiplex formats with specific primers. The PCR reaction was performed for several genes (*speK, speL, speC, speM, speJ, speH, speA, slA, prtF1, speI, spd1, sdn*, and *speB*), and those samples lacking DNA were used as negative controls. The primer sequence of different genes, their amplification length, and gene description are elucidated in **Table 1**.

**Table 1:** Detection of virulence genes primers used in PCR reaction.

Gene	Primer sequence (5′-3′)	Product (bp)	Source or Reference
*speJ*	speJ-F: ATCTTTCATGGGTACG	535	Rato et al., 2011
	speJ-R: TTTCATGTTTATTGCC		
*speH*	speH-F: AGATTGGATATCACAGG	416	Rato et al., 2011
	speH-R: CTATTCTCTCGTTATTGG		
*speI*	speI-F: AATGAAGGTCCGCCATTTTC	516	Rato et al., 2011
	speI-R: TCTCTCTGTCACCATGTCCTG		
*speA*	speA-F: ATGGAAAACAATAAAAAAGTATTG	755	Rato et al., 2011
	speA-R: TTACTTGGTTGTTAGGTAGACTTC		
*Prtf1*	Prtf1-F: TATCAAAATCTTCTAAGTGCTGAG	930	Rato et al., 2011
	Prtf1-R: AATGGAACACTAACTTCGGACGGG		
*sla*	sla-F: CTCTAATAGCATCGGCTACGC	440	Rato et al., 2011
	sla-R: AATGGAAAATGGCACTGAAAG		
*speK*	speK-F: TACAAATGATGTTAGAAATCCAAGGAACATATATGCT	656	Rato et al., 2011
	speK-R: CAAAGTGACTTACTTTACTCATATCAATCGTTTC		
*sdn*	Sdn-F: ACCCCATCGGAAGATAAAGC	489	Rato et al., 2011
	Sdn-R: AACGTTCAACAGGCGCTTAC		
*speL*	speL-F: CTGTTAGGATGGTTTCTGCGGAAGAG	605	Rato et al., 2011
	speL-R: AGCACCTTCCTCTTTCTCGCCT		
*spd1*	spd1-F: CCCTTCAGGATTGCTGTCAT	400	Rato et al., 2011
	spd1-R: ACTGTTGACGCAGCTAGGG		
*speC*	spec-F: GCAGGGTAAATTTTTCAACGACACACA	407	Rato et al., 2011
	spec-R: TGTGCCAATTTCGATTCTGCCGC		
*speM*	speM-F: CCAATATGAAGATAACAAAGAAAATTGGCACCC	600	Rato et al., 2011
	speM-R: CAAAGTGACTTACTTTACTCATATCAATCGTTTC		
*speB*	SpeB-F: ATGAATAAAAAGAAATTAGGTGTCAG	1200	This study
	SpeB-R: CTAAGGTTTGATGCCTACAA		


### Detection of Antibiotic Genes in *S. pyogenes*

To check the presence of antibiotic resistant (genotypes) genes in NBMKU12 isolate, amplification was performed in a single or multiplex PCR with specific primers. The presence of macrolide resistant genes *mef(A)*, tetracycline resistant genes *tet(M), tet(O), tet(Q), tet(T)*, beta-lactam resistant genes *oxa, tem*, chloramphenicol resistant genes *cat1, cmLA*, ampicillin resistant genes *mox1, dha1*, and penicillin resistant genes *pbp1a* and *pbp2b* were tested either by single or multiplex PCR as described in **Table 2**.

**Table 2:** Detection of antibiotic resistance genes primers used in PCR reaction.

Gene	Primer Sequence (5′-3′)	Product (bp)	Source or Reference
*mefA*	mefA-F: GACCAAAAGCCACAATTGTGGA	1432	Pires et al., 2005
	mefA-R: CCTCCTGTCTATAATCGCATG		
*tetM*	tetM-F: TGGAATTGATTTATCAACGG	1080	Pires et al., 2005
	tetM-R: TTCCAACCATACAATCCTTG		
*tetO*	tetO-F: AACTTAGGCATTCTGGCTCAC	515	Ng et al., 2001
	tetO-R: TCCCACTGTTCCATATCGTCA		
*tetT*	tetT-F: AAGGTTTATTATATAAAAGTG	169	Aminov et al., 2001
	tetT-R: AGGTGTATCTATGATATTTAC		
*tetQ*	tetQ-F: TTATACTTCCTCCGGCATCG		
	tetQ-R: ATCGGTTCGAGAATGTCCAC	904	Ng et al., 2001
*Pen PBP1a*	Pen PBP1a-F: CGGCATTCGATTTGATTCGCTTCT	2400	Coffey et al., 1991
	Pen PBP1a-R: CTGAGAAGATGTCTTCTCAGG		
*Pen PBP2B*	Pen PBP2B-F: GATCCTCTAAATGATTCTCAGGTGG	1500	Muñoz et al., 1991
	Pen PBP2B-R: CAATTAGCTTAGCAATAGGTGTTGG		
*Chlor catA1*	Chlor catA1-F: AGTTGCTCAATGTACCTATAACC	547	Van et al., 2008
	Chlor catA1-R: TTGTAATTCATTAAGCATTCTGCC		
*cmlA*	cmlA-F: CCGCCACGGTGTTGTTGTTATC	698	Van et al., 2008
	cmlA-R: CACCTTGCCTGCCCATCATTAG		
*Amp*	Amp mox1-F: GCTGCTCAAGGAGCACAGGAT	520	Van et al., 2008
	Amp mox1-R: CACATTGACATAGGTGTGGTGC		
*Amp*	Amp DHA1-F: AACTTTCACAGGTGTGCTGGGT	405	Van et al., 2008
	Amp DHA1-R: CCGTACGCATACTGGCTTTGC		
*Bla*	Bla OXA-F: GCAGCGCCAGTGCATCAAC	198	Van et al., 2008
	Bla OXA-R: CCGCATCAAATGCCATAAGTG		
*Bla*	Bla TEM-F: GAGTATTCAACATTTTCGT	857	Van et al., 2008
	Bla TEM-R: ACCAATGCTTAATCAGTGA		


### Plate Assay for Lytic Activity in *S. pyogenes*

Cysteine protease activity of *S. pyogenes* NBMKU12 isolate was evaluated by standard casein, papaya, and pineapple (bromelain) hydrolysis with slight modifications (Olsen et al., 2015). Briefly, the isolate NBMKU12 was taken from cryopreserved stocks and inoculated on Columbia agar supplemented with 5% sheep blood (HiMedia, India), and then incubated at 37°C for 24 h. Fresh colonies of NBMKU12 isolate were subcultured for 18–20 h in the early stationary growth phase in Todd-Hewitt broth supplemented with 0.5% yeast extract. A 1.25 mL of early stationary growth culture (5%) was inoculated in 25 mL Todd-Hewitt broth supplemented with 0.5% yeast extract and incubated at 37°C for 24–48 h. The culture was centrifuged and filtered (0.22 μm, HiMedia, India), and then concentrated by lyophilization (Alpha 1-2 LDPlus, Vacuubrand GMBH, Germany). A 200 μL of the concentrated supernatant was added on 1% casein agar, papaya agar, and pineapple agar well plates. The plates were incubated for 24 h at 37°C in an aerobic chamber (Hemco Equipment, India). The digested plates were stained using 1% Congo red staining and further steps followed by Balasubramanian et al. (2012a). Activities of the secreted cysteine protease were studied by measuring the zone of casein, papaya, and pineapple lyses around each well, using a standard ruler scale.

### *speB* Gene Cloning and Sequence Analysis

Based on the *speB* gene sequence available in the GenBank database (NCBI), the specific primers *speB*-F (5′-ATGAATAAAAAGAAATTAGGTGTCAG-3′) and *speB*-R (5′-CTAAGGTTTGATGCCTACAA-3) were designed to amplify the full length gene. The PCR reactions were performed in the following conditions: 95°C for 5 min, followed by 35 cycles at 95°C for 30 s, 45°C for 60 s, and 72°C for 30 s, and a final extension at 72°C for 7 min. The PCR amplification was confirmed by agarose gel electrophoresis (1%), the amplicon cloned in pCR4-TOPO vector (Invitrogen, Germany) and transformed into TOP10 cells by the heat shock method. The DNA insert were conformed by PCR. The DNA was isolated (HiMedia, India) from positive clones, and then sequenced (Macrogen, South Korea). The full-length DNA was obtained by joining the two fragments using the Bio-Edit Program.

### Bioinformatics Analysis

Cysteine protein motifs were analyzed using the following programs: Simple Modular Architecture Research Tool (SMART)^1^, Conserved Domain search from NCBI-CD^2^, signal peptide from Signal lP^3^, and prediction of non-classical protein secretion-SecretomeP^4^. The physico-chemical properties were determined from ProtParam using the ExPASy tool^5^. The sequence similarities were determined from NCBI-BLAST^6^, and a multiple sequence alignment was determined using CLUSTAL Win BioEdit 7.0.

### *In silico* Analysis

The gene sequence encodes for cysteine protease were used for the prediction of 3-dimensional protein structures [3D] by homology modeling using MODELLER 9v7 (Sali and Blundell, 1993). The constructed tertiary structure was validated for quality, with the help of online servers such as PROCHECK (Laskowaski et al., 1993), PROSA (Wiederstein and Sippl, 2007), and VERIFY-3D (Eisenberg et al., 1997). The validated model was studied for the interaction of cysteine protease with different antibiotics, inhibitors, and substrate, by using AutoDock4.0 (Morris et al., 2009) and Patchdock (Schneidman-Duhovny et al., 2005). Visualization of the 3D structure and the study of interaction profiles were carried out with the help of Pymol^7^ and Ligplot (Wallace et al., 1995).

### Secondary Structure Analysis

The secondary structure of cysteine protease was analyzed the Self-Optimized Prediction Method Program (SOPMA) (Geourjon and Deléage, 1995), and its physico-chemical properties were analyzed using ProtParam (Gasteiger et al., 2005).

### Homology Modeling of Cysteine Protease

The suitable template sequence for cysteine protease structure prediction was identified by BLAST program and retrieved from the PDB. The crystal structure of the mature streptococcal Cysteine protease, mSpeB, was used as a template (PDBID: 2UZJ) (Olsen et al., 2009) with a resolution of 1.55 Å. Homology modeling of the cysteine protease was performed using MODELLER 9v7. The model that was constructed with a low molecular objective function (MOF) value was selected and used for docking studies.

### Molecular Docking

The selected 3D models of cysteine protease, antibiotics, inhibitors, and substrate were prepared for molecular docking using the AutoDock tool. Auto Grid (Wiederstein and Sippl, 2007) was used to define the active site. A 41_43_45 points were set as the grid size, with a grid spacing of 0.385 Å. The docked conformation with a low binding energy was selected for further analysis.

## Results

### Bacterial Identification by HiStrep Latex Agglutination and MALTI-TOF-MS

A clinical isolate of NBMKU12 showed clear hemolysis on sheep blood agar and, after further testing with an antiserum grouping HiStrep Latex kit, confirmed agglutination for GAS. In addition, the isolate NBMKU12 suspected of being GAS was identified using MALDI-TOF-MS with m/z score 99.9%. After identification, this strain was labeled as *Streptococcus pyogenes* NBMKU12.

### MIC Test

Based on the CLSI recommendations, the MIC test was carried out for NBMKU12 isolate. The MIC analysis showed antibiotic susceptibilities to ampicillin (0.25 mcg/mL), chloramphenicol (4 mcg/mL), ceftriaxone (1.5 mcg/mL), clavulanic acid (2.5 mcg/mL), and vancomycin (1 mcg/mL). The antibiotic concentrations in the disks were selected based on the CLSI and other published literature information.

### Antibiotic Susceptibility Test

Out of the seven *S. pyogenes* isolates, 25.3% were found to be resistant to multiple antimicrobial agents. The resistance to other antibiotics were observed as follows: ampicillin 71.4%, ceftriaxone 57.1%, and penicillin-G 42.8%. No resistance was observed for the antibiotics amoxiclav, azithromycin, and erythromycin (**Figure 1**).

**FIGURE 1:** Antibiotics susceptibility test in *Streptococcus pyogenes* NBMKU12 isolate. Pen, penicillin; amp, ampicillin; cef, ceftriaxone; chl, chloramphenicol; van, vancomycin; ama, amoxiclav; tet, tetracycline; ery, erythromycin; azy, azithromycin.

### Detection of Virulence Genes in *S. pyogenes*

We screened the isolate NBMKU12 for 13 bacteriophage-associated virulence genes, either pyrogenic exotoxins or superantigens. The screening resulted in the identification of two pyrogenic exotoxin genes, *speJ* and *speB* (**Figure 2**). Of these two, we selected the *speB* gene for further molecular characterization and to encode for a cysteine protease that is involved in host immune suppression.

**FIGURE 2:** Virulence genes detection in *Streptococcus pyogenes* NBMKU12 isolate. M, Marker DNA (100 bp DNA Ladder H3 RTU, GeneDireX), speB amplification (1.2 kb), speJ (535 bp).

### Detection of Antibiotic Genes in *S. pyogenes*

To understand the antibiotic resistance genotype in NBMKU12 isolate, we performed the PCR reaction for 13 antibiotic genes [*mef*(*A*), *tet*(*M*), *tet*(*O*), *tet*(*Q*), *tet*(*T*), *OXA*, *TEM*, *cat1*, *cmlA, mox1, DHA1, PBP1a*, and PBP*2B*] in a single and multiplex PCR. Among these, the Beta lactam (*TEM*) gene was the only gene that was detected in the NBMKU12 isolate (data not shown).

### *speB* Gene Cloning and Sequence Analysis

The NBMKU12 isolate’s *speB* gene cloned full length sequence was obtained by joining the forward and reverse sequences. The full-length gene sequence was deposited in the GenBank database, and an accession number was obtained (MF574208). The *speB* gene consists of 1197 nucleotides with an open reading frame (ORF) of 398 amino acid residues. In this cysteine protease, 1–22 aa is a signal peptide, 22–23 aa is a cleavage site, and 160–367 aa is composed of the catalytic domain. The calculated theoretical pI for cysteine protease is 8.76 and the molecular mass is 43.2 kDa.

The NCBI-BLASTp program revealed that the *speB* putative amino acid sequence of cysteine protease has 99% similarities to *Streptococcus pyogenes* pyrogenic exotoxins B (*speB*), peptidase 10, and streptopain, in different *S. pyogenes* strains as follows*: Streptococcus pyogenes* streptopain (GenBank Accession No. WP_023079791), *Streptococcus pyogenes* streptopain (WP_011285235), *Streptococcus pyogenes* pyrogenic exotoxins B (BAB40954), *Streptococcus pyogenes* pyrogenic exotoxins B (AAA27000), *Streptococcus pyogenes* streptopain (WP_002991253), *Streptococcus pyogenes* streptopain (WP_038433740), *Streptococcus pyogenes* peptidase c10 (WP_009881074), *Streptococcus pyogenes* peptidase c10 (WP_063811911), and *Streptococcus pyogenes* pyrogenic exotoxins B (WP_076639504) (**Figure 3**).

**FIGURE 3:** Alignment of the amino acid sequence of cysteine protease domain from *Streptococcus pyogenes* NBMKU12, with other cysteine proteases from *Streptococcus pyogenes* (WP_023079791), *Streptococcus pyogenes* (WP_011285235), *Streptococcus pyogenes* (ABX44733), *Streptococcus pyogenes* (WP_023610705), *Streptococcus pseudoporcinus* (WP_077322996), *Streptococcus porcinus* (WP_003083607), *Streptococcus didelphis* (WP_018367158). Areas shaded in dark green followed by light green indicates a high degree of similarity (>80%), and unshaded areas are regions of variability among the proteins.

### Plate Assay for Lytic Activity of *S. pyogenes*

The culture supernatant of *S. pyogenes* NBMKU12 was tested, at different durations of incubation, for lysis on 1% casein, papaya, and pineapple (Bromelain) amended agar. The lysis was read as the extent of the clearing zone around the well on the respective agar plates. This lysis is due to the crude concentrated supernatant of *S. pyogenes* NBMKU12, which varied based on the duration of incubation. A large and prominent lysis zone was observed after 24 and 36 h of incubation (**Figure 4**). Among the substrates tested, a large lysis zone was observed on the pineapple agar, followed by one on the papaya agar.

**FIGURE 4:** Cysteine protease hydrolytic activity assay in *Streptococcus pyogenes* NBMKU12 isolate. **(A)** Casein agar, **(B)** Papaya agar, **(C)** Pineapple agar (a: 24 h, b: 36 h, c: 48 h incubated culture filtrates).

### *In silico* Analysis

#### Secondary Structure Analysis

The cysteine protease secondary structure analysis revealed that 33.67, 34.92, 20.60, and 10.80% amino acid residues are present in the form of a helix, random coil, extended strand, and turns, respectively (**Table 3**). The random coil occupies the largest part of the protein, followed by alpha helix, extended strand, and then beta turns. This clearly indicates that the protein is stable. The PsiPred analysis revealed that the cysteine protease consists of 7 Helices, 11 Strands, and 19 Coils (**Figure 5**).

**Table 3:** Secondary structure analysis by PsiPred and SOPMA tool.

S. No.	Structure	Numbers PsiPred	SOPMA (%)
1	Helix	7	33.67
2	Strand	11	20.60
3	Coil	19	34.92
4	Beta turn	–	10.80


**FIGURE 5:** Predicted structure of cysteine protease shows rainbow colored cartoon representation; Helices, Coil and Strands are labeled.

#### Homology Modeling and Validation

The crystal structure of the mature Streptococcal cysteine protease, mSpeB, was used as a template (PDBID: 2UZJ) with the resolution of 1.55 Å. This was selected based on the BLAST result, and the target model (cysteine protease) was built using MODELLER 9v7. Based on the physico-chemical properties of the predicted molecule, the resulting model has four chains (A, B, C, and D) with a molecular weight of 43,204.36 Da and an instability index [II] of 35.20. This classified the protein as a stable protein, and the minimized energy of the molecule was calculated as 79,634.656 kJ/mol.

The PROCHECK analysis of the cysteine protease model showed that 93% of residues were found in the most favored region, 4.9% residues in the allowed regions, and 1.2% residues in generously allowed regions (**Table 4**), which suggests that the model is of good quality. In addition, the PROSA tool (Supplementary Figures 1a,b) shows the *Z*-score of the cysteine protease structure to be -8.3, a value that is within the acceptable range. The atomic model’s (3D) compatibility with its own amino acid sequence (1D) shows a model score of 0.79, which was found to be close to the template score (0.69).

**Table 4:** Stereo-chemical quality of cysteine protease by PROCHECK and model evaluation by PROSA.

PROCHECK			PROSA *Z*-score
	
Favored	Allowed	Outlier	
region (%)	region (%)	region (%)	
93.9	4.9	1.2	-8.3


#### Molecular Docking of Cysteine Protease

The amino acid residues involved in the active site of the cysteine protease are HGEKVSNYAFQLM. The binding affinities of cysteine protease with penicillin-G (**Figure 6A**), erythromycin (**Figure 6B**), azithromycin (**Figure 6C**), and chloramphenicol (**Figure 6D**) are -8.8, -14.8, -15.5, and -13.5, respectively (Supplementary Table 1a). Of these, azithromycin strongly interacts with the receptor in the residue of VAL184 with 2.40 Å length, and the docking happens with inhibitors Cystatin A (**Figure 7A**), Cystatin B (**Figure 7B**), and Cystatin S (**Figure 7C** and Supplementary Table 1b) with the scores of 15194, 18223, and 12115, respectively. Finally, the model was docked with the papain substrate, and the binding score is 17044 (**Figure 7D** and Supplementary Table 1b).

**FIGURE 6:** Docked complex showing interactions between cysteine protease with **(A)** Penicillin-G, **(B)** Azithromycin, **(C)** Erythromycin, **(D)** Chloramphenicol.

**FIGURE 7:** Docked complex showing interactions between cysteine protease and inhibitor **(A)** Cystatin A, **(B)** Cystatin C, **(C)** Cystatin S, **(D)** Papain.

## Discussion

We have used antibody agglutination tests for the identification of streptococcus isolates. Further, the MALTI-TOF-MS has also precisely confirmed that the isolate NBMKU12 belongs to the GAS. Previously, GAS clinical isolates have been identified by MALTI-TOF-MS (Carbonnelle et al., 2011; Peârez-Sancho et al., 2017), and also group B Streptococcus (GBS) (Binghuai et al., 2014; Singhai et al., 2015). The NBMKU12 was isolated from a male patient with a UTI. The streptococcal isolates were characterized by antibiogram assay with nine antibiotics, and the present study focuses on the specific isolate NBMKU12. Antibiogram tests revealed that the isolate NBMKU12 showed 33.3% of resistance. NBMKU12 showed resistance toward ampicillin, penicillin-G, and ceftriaxone, while it showed intermediate resistance (IR) toward tetracycline. However, it was found to be susceptible to amoxiclav, chloramphenicol, erythromycin, azithromycin, and vancomycin. Bacitracin resistance of *S. pyogenes* in Europe was shown to be associated with the cMLSB phenotype-erm(B) genotype described (Silva-Costa et al., 2006). However, the isolates that were susceptible to tetracycline were also reported (Perez-Trallero et al., 2007). Furthermore, 66 Ciprofloxacin resistant isolates of *S. pyogenes* that were collected from infected children (Pires et al., 2010) and *S. pyogenes* isolates with reduced susceptibility to fluoroquinolones (Doloy et al., 2008), or with high-level resistance, have been observed and described earlier (Malhotra-Kumar et al., 2009). In addition, 45 bacitracin-resistant *S. pyogenes* isolates were reported among a batch of 1629 isolates (Pires et al., 2009). These reports have suggested that *S. pyogenes* are becoming resistant to the antibiotics available worldwide.

Based on the present antibiogram study, the NBMKU12 isolate was analyzed for the presence of 13 resistance genes encoding five antibiotics. The result showed the presence of only the Beta-lactem (*TEM*) gene. Although the novel isolate NBMKU12 is phenotypically resistant toward ampicillin and penicillin-G, it shows IR toward tetracycline. However, the mechanism of resistance rendered by these antibiotic resistance genes, is still elusive. Furthermore, the *S. pyogenes* efflux system encoding *mef(A*) gene was also not found. On the other hand, the *bacA* gene encoding bacitracin antibiotic resistance was found in *S. pyogenes* (Chalker et al., 2000). The presence of beta lactamase has been reported as a possible protective mechanism in group A beta hemolytic streptococci (GABHS) (Brook and Gilmore, 1993). Interestingly, we have also found the Beta-lactam resistance gene *TEM* in most of our isolates, including NBMKU12, which indicates its likely role in the resistance to beta-lactam antibiotics.

The streptococcal genes encode exotoxins, superantigens, and streptodornases, which are responsible for GAS virulence and pathogenesis (Igwe et al., 2003; Pires et al., 2009). Most of the diseases caused by GAS are probably due to the diversity of the virulent gene’s products mainly encoded by mobile genetic elements, i.e., prophages (Walker et al., 2014; Kuleshevich et al., 2017). Furthermore, streptococcal pyrogenic exotoxins (s*peA* or *speC*) and streptococcal superantigen (*ssa*) are bacteriophage encoded virulence factors that are associated with invasive diseases (McCormick et al., 2001). Moreover, streptococcal invasion caused by *PrtF1* mediates adherence and internalization by host epithelial cells (Pires et al., 2012). This study analyzed 13 virulent genes of different sizes, and among them streptococcal pyrogenic exotoxins *speJ* and *speB* genes were detected. The *speB* gene encoding for cysteine proteases, which are involved in the host tissue destruction during pathogenesis, was documented (Do et al., 2017).

During infection, GAS secreted cell associated proteins, such as toxins, superantigens, and proteases (Pires et al., 2012; Sumitomo et al., 2013). Despite these virulence factors, the GAS extracellular proteins are important for pathogenesis, especially in epithelial barrier dysfunction (Sumitomo et al., 2013). We have shown the evidence for *speB*, a broad spectrum secreted cysteine protease, which effectively digests cysteine substrates such as casein, papaya, and pineapple (bromelain). The culture supernatant from *S. pyogenes* strains SSI-9 and NZ131 is capable of cleaving the E-cadherin fragment (Sumitomo et al., 2013) whereas, *speB* coding cysteine protease cleaves intercellular junctions, and its proteolytic activity contributes to GAS translocation across the epithelial barrier (Sumitomo et al., 2013). In addition, *speB* extracellular protein of *S. pyogenes* culture supernatant degrades the host extracellular matrix, immunoglobulins, complementary components, and also streptococcal surface proteins (Nelson et al., 2011; Honda-Ogawa et al., 2013). We also noted that the NBMKU12 culture supernatants at different growth periods showed a varied efficiency of digestion of casein, papaya, and pineapple (bromelain) substrates. The cysteine protease secretion into the medium containing the three natural substrates, and their digestion, confirms the presence of predicted signal peptides. On the other hand, aspartic protease sc-asp113 have confirmed the presence of predicted signal peptides in putative protein (Balasubramanian et al., 2012b).

To understand the *speB* encoding cysteine protease interaction in NBMKU12 isolate, the 1.2 kb *speB* gene was amplified, cloned, and the gene sequenced. *S. pyogenes* NBMKU12 was found to be resistant to certain antibiotics. Therefore, to understand the *speB* cysteine protease interaction with commercial antibiotics, inhibitors, and substrates, a docking analysis was performed. The predicted secondary structure of cysteine protease was computed by SOPMA and the results revealed similarity to the model, except the coil region (Dhanavade et al., 2013), and very close to the model of Rana et al. (2017). The major part of the cysteine protein was composed of random coil structure, followed by alpha helix, extended strand, and beta turns structures, and thus the results confirmed the stability of the protein. This computed value is very close to the model of cysteine protease YopT of *Yersinia pestis*, particularly the coil region (Anayet Hasan et al., 2014). The results of PROCHECK, PROSA and VERIFY-3D programs showed the model score to be 0.79, which is close to the template score (0.69). This score is also very close to the cysteine protease YopT of *Yersinia pestis* (Anayet Hasan et al., 2014).

The analysis of the energy profiles of docking conformations of cysteine protease with chloramphenicol, penicillin-G, erythromycin, and azithromycin have showed that erythromycin and azithromycin have lower docking energies. This is because of the existence of an increased number of interactions (Musyoka et al., 2016). Therefore, it can be inferred that erythromycin tightly interacts with cysteine protease resulting in increased stability and reduced flexibility (Siklos et al., 2015). Hence, this drug has higher significance, and azithromycin is placed in the next level of significance. Our wet lab results also infer the same confirmation, where the docking with the inhibitors Cystatin A, Cystatin B, and Cystatin S produce the score 15194, 18223, and 12115, respectively. The GLY 157 of Cystatin A plays a crucial role in the interaction of the inhibitor with cysteine protease, because this residue lies close to the receptor with 2.9 Å bond length and lower binding energy in comparison to other residual interactions. When compared with interaction profiles of azithromycin, this is a higher value, but is closer to the value of papain. The residues TRY67, ASP213, GLY66, and THR215 of cysteine protease interact with ALA2 and ALA3 of the substrate papain residues. Among these residual interactions, THR215 is found to have a short bond length of 2.59 Å. Our laboratory experiments and *in silico* analyses have confirmed the same findings for the isolate NBMKU12. The experimental results confirmed that the isolate NBMKU12 is resistant to penicillin-G and susceptible to erythromycin and azithromycin, followed by chloramphenicol.

## Conclusion

The present study revealed the antibiotic resistant phenotype, genotype, and cloning of *speB* gene encoding cysteine protease and its putative protein interaction with commercially available antibiotics, which are currently being used in the treatment of *streptococcus* infections. Based on the cysteine protease and antibiotic interaction, we confirmed the antibiotic resistance and susceptibility of the isolate NBMKU12. Further investigations must focus on the production and purification of cysteine protease to evaluate the role of *speB* encoding cysteine protease in the pathogenesis of *S. pyogenes* NBMKU12 isolate.

## Author Contributions

NB conducted the experiments, planned and wrote the manuscript. GV conducted the *in silico* analysis. VS helped to perform the experiments and write the manuscript. KB collaborated with the other authors to correct the manuscript. MT provided the sample and collaborated with the other authors to correct the manuscript.

## Conflict of Interest Statement

The authors declare that the research was conducted in the absence of any commercial or financial relationships that could be construed as a potential conflict of interest.

## Footnotes

1 http://smart.embl-heidelberg.de/

2 http://www.ncbi.nlm.nih.gov/Structure/cdd/wrpsb.cgi

3 http://www.cbs.dtu.dk/services/SignalP/

4 http://www.cbs.dtu.dk/services/SecretomeP/

5 http://expasy.org/tools/protparam.html

6 http://www.ncbi.nlm.nih.gov/BLAST/

7 http://PyMOL.sourceforge.net/
